The article "Readiness for Hospital Discharge and Its Correlation with the Quality of Discharge Teaching among the Parents of Premature Infants in NICU" was retracted in 2023. Reasons: signs of a paper mill; suspected computer-generated content; unreliable results or conclusions; lack of ethics approval or compliance.

# Readiness for Hospital Discharge and Its Correlation with the Quality of Discharge Teaching among the Parents of Premature Infants in NICU

**DOI:** 10.1155/2022/4924021

**Published:** 2022-07-13

**Authors:** Li Meng, Zhang Lingling, Zhang Haihong, Zhang Xiaobai, Huang Dandan, Wu Shaoyan

**Affiliations:** ^1^Health Management Center, The First Affiliated Hospital of Chongqing Medical University, Chongqing, 400016, China; ^2^The First Affiliated Hospital and Clinical Medicine College, Henan University of Science and Technology, Luoyang, 471003, China

## Abstract

**Objectives:**

To assess the extent of the readiness for hospital discharge and the correlation with discharge teaching quality among parents of premature infants' in the NICU.

**Background:**

Low readiness for discharge from the hospital can lead to negative outcomes in healthcare for infants born prematurely and their parents. Discharge guidelines are a basic approach to ensure the readiness of the parents for discharge from the hospital. No investigation has ever been conducted into the sufficiency of hospital discharge guidelines for premature infants and their impact on parental readiness for hospital discharge.

**Design:**

Data was collected from four hospitals in China using a correlational descriptive study.

**Methods:**

Two hundred and eight parents of premature NICU-hospitalized infants of four tertiary hospitals in Henan Province from May to October 2020 were enrolled. The general information questionnaire, the readiness for hospital discharge scale- (RHDS-) parent form, and the quality of discharge teaching scale- (QDTS-) parent form were used for data collection. Spearman correlation analysis and descriptive statistics were used to analyze the data.

**Results:**

The total score for hospital discharge readiness was high (8.05 ± 1.11). The total score of the quality of discharge guidelines was moderate (7.44 ± 1.44). Moreover, the discharge teaching quality was positively correlated with the parents' readiness. Positive correlations were found between PRHDS and QDTS subscales, including content received and delivery, physical-emotional status, knowledge, and expected support.

**Conclusion:**

The quality of the discharge guidelines perceived by parents of premature infants was moderate, which may have reduced their readiness for hospital discharge. *Relevance to Clinical Practice*. This study furnishes basic information on the importance of readiness of discharge for the parents of premature infants. The teaching guides nurses to enhance the quality of discharge teaching and the readiness of parents for discharge from the hospital.

## 1. Introduction

Premature infants are newborns whose gestational age was less than 37 weeks (259 days), and their weight was mostly less than 2500 g [1]. According to the latest systematic evaluation report published by the World Health Organization (WHO) in 2019, the global incidence of premature infants was 10.6% on average and was about 6.9% in China [2]. The premature infants' organs were often immature at birth and accompanied by severe comorbidities, such as hypoxic-ischemic encephalopathy, bronchopulmonary dysplasia, respiratory distress syndrome, and apnea, so they were sent to the Neonatal Intensive Care Unit (NICU) after birth for treatment [3]. At present, most NICUs in China are under closed management, so parents have fewer opportunities to contact their children and receive parenting education. As a result, parents of premature infants have been delayed in playing parenting roles. They had insufficient parenting knowledge and lacked proper preparation when premature infants were discharged from the hospital [4]. Premature infants' parents have been shown to be incompetent for home care tasks due to insufficient readiness for hospital discharge, resulting in unhealthy emotions such as tension and anxiety [5]. In addition, parents were unable to provide good care for premature infants, which resulted in growth retardation of premature infants, high readmission rates, and so on [6, 7]. Therefore, improving the readiness for discharge from the hospital was advantageous to improve the psychological condition of the parents and ensure the safety of home care for preterm infants.

Currently, clinicians use a set of clinical criteria to determine whether or not a premature infant is ready for discharge from the hospital. Family members and healthcare providers may have different assessments of a patient's readiness for discharge, according to research [8, 9]. Few resources are available to help parents of premature infants get ready for their children's discharge from the hospital. To better meet the needs of families with premature infants, it is essential to create an instrument that can accurately assess whether or not they are prepared for their infant's discharge from the NICU.

Discharge teaching means that medical staff convey medical information to premature infants' parents in the form of education or communication. It can provide parents with postdischarge care methods, related precautions, medication, rehabilitation training, and other medical care information. The guidance skills will affect the parents' understanding, acceptance, and correct implementation of the content. High-quality discharge teaching provided by nurses is an essential element of this smooth transition and would assist parents in preparing for the discharge of their preterm infant. High-quality discharge education can improve parents' readiness for hospital discharge, which ultimately enhances the cure rate and prevents complications [10–12]. However, few literature or reports have investigated the current status of discharge teaching quality for premature infants' parents and its relationship with hospital discharge readiness. Thus, this study is aimed at understanding the current status of readiness of the parents and the quality of discharge guide when premature infants were discharged from the hospital and at assessing the association between the readiness for discharge from the hospital and the quality of teaching for the same, to provide references for future intervention studies and other related studies to enhance the readiness of the parents of premature infants.

### 1.1. Background

The readiness for hospital discharge (RHD) and the quality of discharge teaching (QDT) are two leading indicators used to assess the quality of discharge services [13]. It has been said that RHD is a multifactored concept that provides an estimate of a patient's potential to be discharged from an acute care facility [14]. The parents of a hospitalized child face special difficulties as they prepare for their child's discharge. Because children have age-related vulnerabilities that require special planning and selection of resources for their medical and developmental needs, the age of the child may affect parental readiness [15]. Parental and infant demographics, hospitalization factors, and nursing practice variables have all been examined in the context of predicting parental readiness. Only the presence of additional children and the effectiveness of discharge education were found to be consistently significant predictors of parental readiness [16]. Teaching is the primary method that nurses use to prepare patients and their families for discharge and the transition home from the hospital [17]. Readmissions and emergency visits can be decreased by providing a consistent transition from the hospital to the patient's home [18].

Several measures have been developed to assess patients' or caregivers' readiness for hospital discharge, including the PREPARED Questionnaire [19], the Care Transitions Measure (CTM) [20], the Readiness for Discharge Questionnaire (RDQ) [21], the Post Anesthetic Discharge Scoring System (PADSS) [22], and the RHD Scale (RHDS)–Parent Form [23, 24]. The RDQ was created to evaluate the readiness of patients with schizophrenia for discharge, while the PADSS was designed to evaluate postanesthesia recovery. On the day of a patient's discharge, health care providers complete both the RDQ and the PADSS. None of these four measures was intended to assess parental readiness for the discharge of their hospitalized children, despite their excellent reliability and validity.

The literature describes a variety of structural and procedural factors and their effects on patient discharge preparation. The quality of patient-reported discharge teaching and the frequency of readmissions were positively correlated with the number of hours that nurses were available to patients during hospitalization, as shown by Weiss et al. (2011). With increased care time per patient per day, nurses can devote more time to time-consuming tasks such as discharge preparation [25].

However, few studies or reports have examined the current status of discharge teaching quality for parents of premature infants and its relationship to hospital discharge readiness. Therefore, the purpose of this study was to gain an understanding of the current status of the readiness of the parents and the quality of the discharge guide when premature infants were discharged from the hospital, as well as to evaluate the association between the readiness for discharge from the hospital and the quality of teaching for the same, with the end goal of providing references for future intervention investigations and other relevant studies to improve the readiness of the parents of premature infants.

## 2. Methods

### 2.1. Study Setting, Design, and Sampling

A correlational descriptive study was conducted in four tertiary hospitals' neonatal intensive care unit in Henan, China. Selection of samples was done according to eligible criteria for inclusion: premature infants (a) gestational age < 37 weeks (259 days), and moved into NICU after birth; (b) hospitalization time ≥ 3 days, discharge according to doctor's advice; and (c) home as the children's destination after discharge. Parents were (a) adult (≥18 years) with at least elementary school education and above; (b) parents were the main caregivers of premature infants after discharge from the hospital, and their weekly contact time with premature infants was greater than 72 hours. Exclusion criteria included (a) parents of abandoned, readmitted, or deceased premature infants; (b) cognitive skills not sufficient to independently fulfil the questionnaire and consent processes. In the analysis of statistical variables, it is stipulated that for the study of influencing factors, the sample size should be a minimum of 5-10 times the variable number. The maximum number of entries in the scale in this study was 22. Allowing for 20% invalid questionnaires, the estimated range of sample size should be 132 to 264. In this study, 208 parents were invited for participation.

### 2.2. Instruments

This study employed the RHDS-parent form, the demographic form, and the QDT scale (QDTS) parent form as its instruments. Each instrument is detailed herein.

#### 2.2.1. Demographic Form

The demographic form included information about parents, such as their level of education, gender, age, occupation, whether they have received parenting education, experience caring for premature infants, health status, and type of childbirth.

#### 2.2.2. The RHDS-Parent Form

This form was used to assess the perceptions of hospitalized children's parents regarding their readiness for discharge. Wild et al. translated it into Chinese in 2017 in accordance with the international instrument translation guideline [26]. The RHDS-parent form consists of 22 items distributed across four primary subscales: pain status, physical-emotional status, knowledge, and solicited support. The first item on the scale was a true-false question that did not contribute to the overall score. Other items were assigned a score between 0 and 10 points (“complete” to “incomplete”). The RHDS-parent form score ranged between 0 and 220. A greater total score indicated that the parents were more prepared for hospital discharge. Using Cronbach's alpha coefficient, we then evaluated the internal consistency of the reliability of the Chinese version of instruments, obtaining RHDS parent form values for the entire 0.91 scale.

#### 2.2.3. The QDTS-Parent Form

This form was used to evaluate the perspectives of hospitalized children's parents regarding the quality of discharge teaching. There was no Chinese translation available for QDTS-parent form. Chen and Bai translated the RHDS-parent form into Chinese in 2017 in accordance with the instrument translation guideline [9]. This scale consisted of received content and subscale of delivery, with six paired items indicating the quantity of content received and required during discharge preparation. The subscale of delivery, which consisted of 12 items, reflected the teaching abilities of the nurses. The QDTS-parent form utilized a Likert rating scale. The parents responded to each question on the QDTS-parent form with a score between 0 (not at all) and 10 (totally). All of the QDTS-parent form scores were added to the content received and delivery scores, which range from 0 to 180, excluding any content that was required for the total scale score. A higher total score indicates better overall discharge teaching. We then examined the dependability of the Chinese format of instruments for internal consistency using Cronbach's alpha coefficient, obtaining QDTS-parent form values on a complete scale of 0.82.

In the RHDS and QDTS, each measure was categorized and interpreted according to four levels: <7 (low), 7-7.9 (moderate), 8-8.9 (high), and 9-10 (very high) [27].

### 2.3. Ethical Consideration

The permissions for the study were granted by the Research Ethics Committees of one university and four hospitals chosen for the study. One researcher explained the purpose, methodology, and anticipated risks and benefits of this study to the participants. The participants could freely withdraw at any time of the study, without any negative outcomes, and were assured of confidentiality of the study questionnaires and all collected data, as they were numbered with no names.

### 2.4. Process of Data Collection

Entrusted 1-2 nurses from the NICU in each hospital to assist in the investigation, and the researcher conducted unified training for them. Before the premature infants were discharged from the hospital, each participant was provided with a package containing a self-reported questionnaire comprising the QDTS, demographic form, and RHDS. The researcher conducted interviews with the participants who had difficulty completing the questionnaire. The researcher distributed the questionnaires on-site and collected them after completion. In this survey, 240 questionnaires were distributed; 32 questionnaires with missing items or obvious logical errors were eliminated, leaving 208 valid questionnaires.

### 2.5. Analysis of Data

The data were entered using Epidata 3.1 and assessed using SPSS v20.0, including inferential and descriptive statistics. The data on demography and parents' level of perception towards the readiness for discharge from hospital and the status of discharge guidelines were described by describing the minimum and maximum value, standard deviation, the mean, range, and percentage. The Pearson correlation test was used to examine the relationship between hospital readiness and the value of discharge teaching for parents of premature infants.

## 3. Results

### 3.1. Demographic Data of Participants

The mean age of the participating 208 parents of premature infants was 30.13 years (SD = 4.56). Most of them were fathers (62.0%) and mothers (38.0%) and had completed primary school education (2.9%). They had previously worked as workers (68.8%) or farmers (6.7%). Some parents had learned about parenting skills (42.8%). Although only a few participants had prior experience caring for premature infants (7.7%). Almost all of the participants were in good health (95.2%). Over half of premature infants were born by cesarean section (62.5%). The majority of premature infants returned home and were cared for by their parents and other individuals (73.6%; Table 1).

### 3.2. The Readiness for Discharge from Hospital, as Discerned by Premature Infants' Parents

A high overall readiness for hospital discharge was perceived (8.05 ± 1.11). Among the four primary subscales, the knowledge subscale was the lowest (6.91 ± 1.79), both physical-emotional status (8.81 ± 1.01) and expected support subscales (8.69 ± 1.38) were at a high level, and the subscale of pain status was very high (9.27 ± 0.99; Table 2).

### 3.3. The Status of Discharge Guidelines Discerned by Premature Infants' Parents

In accordance with the aforementioned criteria that categorizes the quality of discharge teaching into four grades, Table 3 demonstrates that participants rated the quality of discharge teaching as moderate (7.44 ± 1.44) for content discerned and delivery subscales (7.60 ± 1.46 and 7.12 ± 1.93), but as high (8.50 ± 1.31) for content needed.

### 3.4. The Relationship between Hospital Discharge Readiness and Discharge Guideline Quality among Premature Infants' Parents

The results revealed a positive association between the discharge guideline quality and discharge readiness among premature infants' parents (*r* = 0.448, *P* < 0.01). Moreover, a positive relationship was found between every subscales of the discharge teaching quality and some subscales of the discharge readiness (Table 4).

## 4. Discussion

### 4.1. Hospital Discharge Readiness

The success rate of treatment for premature infants has grown in recent years with the advancement of medical technology. However, premature infants still needed the meticulous care of their parents after they were successfully treated and returned home. Parents are the main caregivers for premature infants after they are discharged from the hospital. If the parents with inadequate readiness for hospital discharge are not well prepared for their emotional and physical status, the insufficient knowledge about care of diseases and the less support available will increase the risk of readmission of premature infants after discharge [28].

Overall, parents of premature infants exhibited a high level of readiness for discharge from the hospital. Pain status, physical-emotional status, expected support, and knowledge were perceived at varying levels, in descending order of score. Only the knowledge subscale was at a low level, whereas all others were at a high or very high level. Consequently, the majority of parents of premature infants adequately prepared their children for the transition from the hospital to their homes, and parents received the expected level of support. This finding is consistent with a previous investigation [29, 30]. This result could arise for several reasons. First, in this study, most families with premature infants had elderly or social childcare institutions to help them care for the children. The study shows that good family and social support could reduce the care burden of those parents [31, 32]. Second, in this research, the age of participating parents ranges from 18 to 45 years old. They had a strong ability to use the Internet, and they think that they can quickly obtain the corresponding parenting knowledge through parenting-related WeChat public accounts, software, etc., which enhances their confidence in caring for the children. Third, 63.5% of parents had not seen their children while they were hospitalized, and they were excited on the day of discharge, when they carried their children home. This could lead to the parents overestimating their readiness for hospital discharge.

### 4.2. The Quality of Guidelines for the Discharge

The quality of guidelines for the discharge discerned by premature infants' parents was moderate, with a lower score of content received than that needed. This is congruent with findings published in earlier studies [33]. This may be related to several reasons. First of all, most of the parents in this study were parents who had their first-born (57.7%), and most of them (57.2%) had not learned parenting knowledge. Therefore, parents of premature infants lacked relevant parenting knowledge and experience. It is anticipated that the pediatric nurse will provide the necessary information about infant care through the teaching process [34]. In other words, parents of premature infants had greater expectations for nurses' discharge instruction. In addition, during the COVID-19 epidemic, the majority of NICUs in China restricted or banned visits. The NICUs of the four hospitals surveyed for this study had almost completely suspended all visits. Thus, premature infants' parents had limited contact with nurses. The education and guidance were only provided to parents on the day of hospitalization. Therefore, parents of premature infants may not have received adequate discharge guidelines from the nurses due to time constraints. In addition, the educational level and medical knowledge of the parents and nurses were unequal, resulting in a lack of understanding and acceptance of medical information by the parents of premature infants. In addition, on the day of discharge, the parents' excitement and anxiety will have a limited impact on the educational effect.

Therefore, nurses should have an adequate understanding of each parent of premature infants and their needs when they provide discharge teaching and use some instructional skills to improve the effectiveness of discharge teaching. In addition, under the NICU closed management mode, the nursing staff should actively choose a variety of discharge teaching forms, such as increasing health education time, implementing early and timely discharge teaching, and expanding the form of health education by utilizing WeChat, the Internet, and other means to provide health education.

### 4.3. The Relationship between the Quality of Discharge Guidelines and Readiness for Discharge among Premature Infants' Parents

According to earlier studies, the correlation between the quality of discharge guidelines and the discharge readiness of parents of premature infants was significantly positive [35, 36]. High-quality discharge teaching is conducive to enhancing parents' ability to care for their children, reducing the uncertainty of illness, and improving their perception of readiness for discharge [37]. Thus, nurses should pay attention to the discharge teaching for parents of premature infants, fully understand the difference between the received and the required content of discharge guidelines for the parents, and provide targeted information to support them according to their individual needs. In the meantime, nurses should also give importance to enhancing knowledge transfer skills, improving the quality of discharge teaching, and then improving parents of premature infants' readiness for hospital discharge in order to ensure the safety of home care for premature infants.

### 4.4. Study Limitations and Strength

The study had several strengths, including an adequate sample size, which allowed for a sufficient analysis of the quality and readiness of the discharge guidelines. We collected data from four hospitals, and it can be generally applied to other hospitals in China. The current study instruments were designed to generate essential, specific content for parents of premature infants, and their authenticity and content validity were acceptable. However, the use of a convenience sampling method during data collection was a limitation of this study.

## 5. Conclusions

In conclusion, a correlation was found between the quality of hospital discharge guidelines and readiness for hospital discharge. However, participants perceived the discharge guideline quality to be moderate, and the content received by premature infants' parents was insufficient to meet their needs. Therefore, more attention must be paid to the content and methods of delivery of guidelines, and the individual needs of parents and their mastery of discharge teaching content must be understood in order to specifically address the needs of parents' learning while preparing the discharge, thereby enhancing the readiness of premature infants for hospital discharge.

## Figures and Tables

**Table 1:** Demographic data of parents of premature infants (*N* = 208).

Characteristics	Group	*n*	%
Age (years)	18-25	30	14.4
	26-35	157	75.5
	>35	21	10.1
Gender	Father	129	62.0
	Mother	79	38.0
Level of education	Primary school	6	2.9
	Secondary school	108	51.9
	College/university	94	45.2
Occupation	Worker	143	68.8
	Farmer	14	6.7
	Unemployed	34	16.3
	Other	17	8.2
Learning parenting knowledge	Yes	89	42.8
	No	119	57.2
Experience in nursing premature infants	Yes	16	7.7
	No	192	92.3
Health status	Healthy	198	95.2
	General	10	4.8
Delivery method	Vaginal delivery	78	37.5
	Cesarean section	130	62.5
Care type of premature infants	Parents independent care	55	26.4
	Dependent	153	73.6
Visited your child during the hospitalization	Yes	132	63.5
	No	76	36.5

**Table 2:** Perception level of premature infants' parents towards the readiness for discharge from the hospital (*N* = 208).

Readiness scale of parents for discharge from hospital	Items	Mean ± SD	Level
Knowledge subscale	9	6.91 ± 1.79	Low
Taking care of the child		7.05 ± 2.20	
Child's personal needs		7.55 ± 2.08	
Child's growth and development needs		6.72 ± 2.27	
Medical needs		5.97 ± 2.56	
Things to pay attention to after going home		6.78 ± 2.32	
Who and when to call for assistance		8.42 ± 2.20	
What can the child do after returning home		7.25 ± 2.18	
Follow-up treatment		6.03 ± 2.64	
Community medical service		6.41 ± 2.81	
Physical-emotional status subscale	7	8.81 ± 1.01	High
Child's physical readiness		8.65 ± 1.34	
Parent's strength		8.85 ± 1.71	
Child's strength		7.75 ± 1.94	
Mental state of the parents		9.14 ± 1.36	
Mental state of the child		8.21 ± 1.71	
Parent's emotionally ready		9.39 ± 1.18	
Parent's physical fitness		9.67 ± 0.75	
Expected support subscale	4	8.69 ± 1.38	High
Emotional support		9.07 ± 1.28	
Child care support		8.80 ± 1.64	
Household activity support		8.75 ± 1.82	
Medical care or resources support		8.13 ± 2.19	
Pain status subscale	2	9.27 ± 0.99	Very high
Parent's pain		9.86 ± 0.59	
Child's pain		8.68 ± 1.73	
Total scale	22	8.05 ± 1.11	High

**Table 3:** Premature infants' parents' perception of parents of towards the discharge guidelines quality (*N* = 208).

Parents' discharge guideline scale	Items	Mean ± SD	Level
Subscale of needed content	6	8.50 ± 1.31	High
Child's care		8.75 ± 1.69	
Parents' emotions		8.22 ± 2.22	
Medical requirements and treatment		8.84 ± 1.62	
Treatment or medication practice		8.09 ± 2.20	
Person and time to call for assistance		8.64 ± 1.67	
Information for family members		8.46 ± 1.51	
Content received subscale	6	7.12 ± 1.93	Moderate
Child's care		7.41 ± 2.34	
Parents' emotions		6.77 ± 2.79	
Medical needs and treatment		8.18 ± 2.20	
Treatment or medication practice		5.14 ± 3.52	
Who and when to call for assistance		8.02 ± 2.37	
Information for family members		7.22 ± 2.40	
Subscale of delivery	12	7.60 ± 1.46	Moderate
Resolving concerns and questions		8.00 ± 1.96	
Listening to your worries		6.42 ± 2.93	
Paying attention to beliefs and values		5.01 ± 3.38	
Guides the way of caring for children		7.78 ± 2.04	
Teaching in a way could be understood		7.99 ± 2.04	
Understand relevant information providing consistent information		8.04 ± 2.04	
At a good time to guidance		8.88 ± 1.34	
		8.19 ± 1.68	
Family members participate		7.47 ± 2.35	
Enhancing confidence for child care		8.09 ± 1.71	
Knowledge of actions to be performed in an emergency		6.93 ± 2.06	
Reducing anxiousness about returning home		8.35 ± 1.58	
Total scale	18	7.44 ± 1.44	Moderate

**Table 4:** Coefficient for the correlation between the discharge instructions quality and readiness for discharge from the hospital among premature infants' parents (*N* = 208).

Variables	Total readiness for hospital discharge scale	Knowledge	Physical-emotional status	Expected support	Pain status
Total quality of discharge teaching scale	0.448^∗∗^	0.367^∗∗^	0.406^∗∗^	0.354^∗∗^	0.090
Content needed	0.234^∗∗^	0.060	0.379^∗∗^	0.330^∗∗^	0.120
Content received	0.427^∗∗^	0.374^∗∗^	0.337^∗∗^	0.332^∗∗^	0.093
Delivery	0.382^∗∗^	0.297^∗∗^	0.379^∗∗^	0.306^∗∗^	0.073

^∗∗^ *P* < 0.01.

## Data Availability

Data will be provided upon request to the authors.
